The article "SLCO4A1-AS1 mediates pancreatic cancer development via miR-4673/KIF21B axis" was retracted in 2023. Reasons: duplicated images; signs of a paper mill; concerns about the data; concerns about the images.

# SLCO4A1-AS1 mediates pancreatic cancer development via miR-4673/KIF21B axis

**DOI:** 10.1515/med-2022-0418

**Published:** 2022-02-14

**Authors:** Jianxin Zhang, Yanbing Shen, Dandan Ma, Zhonghu Li, Zhiyong Zhang, Weidong Jin

**Affiliations:** Department of General Surgery, General Hospital of Central Theater Command, Wuhan 430070, Hubei, China; Department of General Surgery, General Hospital of Central Theater Command, 627 Wuluo Road, Wuchang District, Wuhan 430070, Hubei, China

**Keywords:** SLCO4A1-AS1, miR-4673, KIF21B, pancreatic cancer

## Abstract

In this study, we intended to figure out the biological significance of long non-coding RNAs (lncRNAs) solute carrier organic anion transporter family member 4A1 antisense RNA 1 (SLCO4A1-AS1) in pancreatic cancer (PC). Cell counting kit-8, colony formation, wound healing, transwell, and flow cytometry experiments were performed to reveal how SLCO4A1-AS1 influences PC cell proliferation, migration, invasion, and apoptosis. Thereafter, bioinformatics analysis, RNA immunoprecipitation assay, luciferase reporter assay, and RNA pull-down assay were applied for determining the binding sites and binding capacities between SLCO4A1-AS1 and miR-4673 or kinesin family member 21B (KIF21B) and miR-4673. The results depicted that SLCO4A1-AS1 was upregulated in PC, and SLCO4A1-AS1 knockdown suppressed PC cell growth, migration, invasion, and induced cell apoptosis. Furthermore, SLCO4A1-AS1 was verified to modulate the expression of KIF21B by binding with miR-4673. SLCO4A1-AS1 exerted an oncogenic function in PC. The overexpression of SLCO4A1-AS1 aggravated the malignant behaviors of PC via the upregulation of KIF21B by sponging miR-4673. Our findings revealed a novel molecular mechanism mediated by SLCO4A1-AS1, which might play a significant role in modulating the biological processes of PC.

## 1 Introduction

Pancreatic cancer (PC) is known as a prevailing malignancy in digestive system worldwide, accounting for approximately 56,770 new cases and 45,750 deaths in America in 2019 [1]. Due to the aggressive malignant behaviors at early stage, the shortage of early diagnostic markers, the lack of effective therapeutic strategies, and the speedy disease progression, the prognosis of patients with PC is extremely unsatisfactory [2,3]. Surgical resection and systemic chemo-radiotherapy are considered as the primary choices for PC treatment [4]. Despite great advances and innovations during the past decades [5,6], the underlying mechanisms of the initiation and progression of PC remain obscure. Therefore, it is urgent to develop a further understanding of the molecular mechanisms underlying PC and identify novel effective biomarkers of PC.

Accumulating evidence has suggested that long non-coding RNAs (lncRNAs) are a type of RNA transcripts in eukaryotic cells longer than 200 nucleotides defined by a lack of protein-coding potential [7]. More and more studies have revealed the regulation of lncRNAs in a range of biological processes, involving cell growth, apoptosis, migration, and invasion in almost all human cancers, including gastric cancer, hepatocellular carcinoma, and prostate cancer [8,9,10,11]. LncRNA solute carrier organic anion transporter family member 4A1 antisense RNA 1 (SLCO4A1-AS1) was verified to be an oncogene in some cancers [12]. For example, in non-small-cell lung cancer, SLCO4A1-AS1 facilitates cellular processes by mediating the miR-223-3p/IKKα/NF-κB signaling [13]. In colorectal cancer, SLCO4A1-AS1 accelerates cell growth and migration via β-catenin-dependent Wnt pathway [14]. SLCO4A1-AS1 binds with miR-335-5p to elevate organic cation/carnitine transporter4 (OCT4) expression, thus aggravating malignant phenotypes of bladder cancer [15]. The GEPIA database indicates that SLCO4A1-AS1 is upregulated in 179 pancreatic adenocarcinoma (PAAD) tissue samples compared with 171 non-tumor tissue samples. Nevertheless, the function and underlying mechanism of SLCO4A1-AS1 in PC remain unclear.

Therefore, this study investigated the regulatory mechanism of SLCO4A1-AS1 in PC cells. Additionally, the role of the SLCO4A1-AS1/miR-4673/KIF21B regulatory network in the malignant progression of PC was explored, providing a better understanding of the pathogenesis of PC.

## 2 Materials and methods

### 2.1 Cell culture

PC cell lines (CAPAN-1, SW1990, CFPAC-1, and Panc 03.27) and human pancreatic duct epithelial cell line (H6C7) used in the study were purchased from American Type Culture Collection (ATCC, Manassas, VA, USA). SW1990 and CAPAN-1 cells were incubated in Dulbecco’s Modified Eagle’s Medium (DMEM; Gibco, NY, USA) containing 10% fetal bovine serum (FBS, Gibco), and Panc 03.27, CFPAC-1, and H6C7 cells were incubated in RPMI 1640 medium containing 10% FBS (Gibco). All cells were maintained at 37°C in a humidified atmosphere with 5% CO_2_.

### 2.2 Cell transfection

Short-hairpin RNAs (shRNAs) for the knockdown of SLCO4A1-AS1 (sh-SLCO4A1-AS1#1/2) were constructed by GenePharma (Shanghai, China), with sh-NC as the negative control (NC). To upregulate SLCO4A1-AS1 and KIF21B, pcDNA3.1/SLCO4A1-AS1 and pcDNA3.1/KIF21B were obtained from GenePharma, respectively. The empty pcDNA3.1 plasmid was regarded as NC. Meanwhile, miR-4673 mimics, miR-4673 inhibitors, and the negative control (NC mimics and NC inhibitors) were synthesized by Thermo Fisher Scientific (Carlsbad, CA, USA). Cell transfection was conducted utilizing Lipofectamine 3000 (Invitrogen, Carlsbad, CA, USA) for 24 h according to the specification of the manufacturer.

### 2.3 Quantitative real-time PCR (qRT-PCR)

Total RNA was isolated and extracted from treated PC cells using TRIzol Reagent (Invitrogen) under the guidelines of the manufacturer. Moreover, complementary DNA (cDNA) was obtained by reverse transcription with extracted RNA using PrimeScript RT Reagent Kit (Invitrogen). Later, qRT-PCR was carried out with SYBR Green PCR Kit (Takara, Dalian, China) on ABI 7500 Fast Real-Time PCR system (Applied Biosystems, Foster City, CA, USA) with particular primers according to the recommendations of the manufacturer. GAPDH and U6 served as the internal controls. The relative expression of RNAs was quantified and analyzed with the 2^−ΔΔCt^ method. Primer sequences are listed in supplementary Table 1.

**Table 1:** Primer sequences used for qRT-PCR

Gene	Sequence (5′ → 3′)
SLCO4A1-AS1	CTGGGCTGACAAGTGAGGAG
SLCO4A1-AS1	GGGTTCAAGTCAGCGACACT
miR-4673	ACACTCCAGCTGGGTCCAGGCAGGAGCCGG
miR-4673	TGGTGTCGTGGAGTCG
miR-7855-5p	ACACTCCAGCTGGGTTGGTGAGGACCCCAA
miR-7855-5p	TGGTGTCGTGGAGTCG
miR-876-3p	CTGTGGTGGTTTACAAAGTAATT
miR-876-3p	GTGCAGGGTCCGAGGT
miR-6783-3p	ACACTCCAGCTGGGTTCCTGGGCTTCTCCT
miR-6783-3p	TGGTGTCGTGGAGTCG
miR-6514-3p	ACACTCCAGCTGGGCTGCCTGTTCTTCCA
miR-6514-3p	TGGTGTCGTGGAGTCG
miR-5001-3p	ACACTCCAGCTGGGTTCTGCCTCTGTCCAG
miR-5001-3p	TGGTGTCGTGGAGTCG
FBXL18	GATGATGACATGCACCCTGC
FBXL18	AGCTGCCTCACTTTGTCCTC
GPR37L1	TCTTGCTGTGATTTTGGCTGTG
GPR37L1	CTCTTGGATCGGCTCTGCTG
CACNG8	ATCATTTCCCGGAGGACACG
CACNG8	CGCCGAAGTAGAAGGACCAG
KIAA1614	CAGCATGAAGCATGGGCATC
KIAA1614	GGTGCTCATACCAGGCACTT
KREMEN1	ACAGTCTGAAATACCCCAACG
KREMEN1	GTTTCCATGATCCTTGTAGCAG
CYB561A3	CACTTCGTCCCACTGTGGTT
CYB561A3	AGGAGGAAGACAGCAAAGCC
KIF21B	ACAGCGACTCCTCTTTGTCG
KIF21B	TTGTGCGCATTGGGGATTTG
AP5S1	AACTACAACCCCCGAAGTGC
AP5S1	ATCAGAGCTGCTGGGTAGGA
GAPDH forward	TATGATGATATCAAGAGGGTAGT
GAPDH reverse	TGTATCCAAACTCATTGTCATAC
U6 forward	CTCGCTTCGGCAGCACA
U6 reverse	AACGCTTCACGAATTTGCGT

### 2.4 Cell counting kit-8 (CCK-8) assay

Cell viability was assessed by CCK-8 assay. Briefly, cells were seeded into 96-well plates (1 × 10^4^ cells/well). Each well was added with 200 µL medium containing CCK-8 reagent (Beyotime, Shanghai, China) after incubation for 0, 24, 48, 72, and 96 h, as instructed by the manufacturer. Next, a microplate reader (Thermo Fisher Scientific) was used for detecting the absorbance at 450 nm of each well.

### 2.5 Colony formation assay

For detecting cell proliferation, transfected PC cells were seeded in 6-well plates (1 × 10^3^ cells/well), followed by 2-week incubation in DMEM containing 10% FBS. Thereafter, cells were stained with crystal violet (Sigma-Aldrich St. Louis, MO, USA) for 30 min after mounted with paraformaldehyde (Sigma-Aldrich) for 15 min. Colony numbers were calculated and analyzed after imaged with a microscope (Olympus, Tokyo, Japan).

### 2.6 Flow cytometry analysis

Flow cytometry was performed to examine cell apoptosis with the utilization of Annexin V-FITC/PI Apoptosis Detection Kit (KeyGEN, Nanjing, China). The harvested cells were suspended in binding buffer and dyed with annexin V-Fluorescein Isothiocyanate (V-FITC) solution and propidium iodide (PI) solution for 15 min. Subsequently, a flow cytometer AccuriC6 (BD Biosciences, Franklin Lakes, NJ, USA) was utilized to observe the dyed cells.

### 2.7 Western blot analysis

48 h after transfection, aggregate proteins were lysed from PC cells utilizing RNA immunoprecipitation assay (RIPA) buffer (Beyotime). Equal amounts of proteins were loaded and segregated via 10% sodium dodecyl sulfate polyacrylamide gel electrophoresis (SDS-PAGE), followed by transferring to polyvinylidene fluoride (PVDF) membranes (Millipore, Boston, MA, USA). Later, the PVDF membranes were blocked with 5% non-fat milk for 2 h, and then incubated with primary antibodies overnight at 4°C, including anti-Bcl-2 (1:2,000, ab182858, Abcam), anti-Bax (1:2,000, ab182733, Abcam), and anti-GAPDH (1:10,000, ab181603, Abcam). Then, after washing three times with Tris-buffered saline with Tween-20 buffer, the membranes were incubated with HRP-conjugated secondary antibodies at room temperature for 2 h. GAPDH served as a loading control. The bands were analyzed using ECL detection system (Thermo Fisher Scientific).

### 2.8 Wound healing assay

The migratory capacity of the transfected PC cells was determined by wound healing assay. Briefly, cells were implanted into 6-well plates until 80% confluence. Then, a 10 µL pipette tip was applied to scratch a straight line in the center of the plates. Besides, the plates were cleaned three times using phosphate-buffered saline to remove cell debris. Subsequently, the cells were incubated in RPMI 1640 medium without serum for another 24 h. Finally, the recovery state of the wounds at 0 and 24 h was observed under a light microscope (Olympus).

### 2.9 Transwell invasion assay

After transfection, PC cells were resuspended in serum-free DMEM and plated into the upper chamber of 24-well transwell (pore size 8 µm; Corning Costar) coated with Matrigel (BD Biosciences). The lower chamber was filled with DMEM containing 10% FBS. After incubation for 24 h, noninvaded cells were removed with cotton swabs, while invaded cells were fixed with 4% paraformaldehyde, and then stained with 0.1% crystal violet for 20 min. The invaded cells were imaged with an inverted microscope (Olympus).

### 2.10 Subcellular fractionation assay

According to the recommendations of the manufacturer, a PARIS™ Kit (Invitrogen) was employed to perform the subcellular fractionation assay. SW1990 and CAPAN-1 cell lines placed into cell fractionation buffer were subjected to centrifugation. Moreover, the supernatant was collected, and the remaining lysates were rinsed with cell fractionation buffer. Next cell nuclei were lysed by cell disruption buffer. Thereafter, the lysate was incubated with the supernatant, ethanol, and 2 × lysis/binding solution. Lastly, cytoplasmic and nuclear RNAs were investigated through qRT-PCR.

### 2.11 Bioinformatics analysis

SLCO4A1-AS1 expression profile in PAAD is shown at GEPIA database (http://gepia.cancer-pku.cn/detail.php? gene=&clicktag=boxplot). This dataset contains 179 PAAD samples and 171 normal samples. DIANA tools – LncBase Predicted v2 (http://carolina.imis.athena-innovation.gr/diana_tools/web/index.php?r=lncbasev2%2Findex) [16] was applied to search for downstream miRNAs of SLCO4A1-AS1 with the screening condition of binding score more than 0.85 and predict the binding site between SLCO4A1-AS1 and miR-4673. After screening out the target gene of miR-4673 with the screening condition of cumulative weighted context^++^ score > −0.86, the binding site between miR-4673 and KIF21B was analyzed with the utilization of TargetScan database (http://www.targetscan.org/vert_71/) [17].

### 2.12 RNA pull-down assay

Biotinylated SLCO4A1-AS1 and a control probe purchased from Genechem Biotech (Shanghai, China) were transfected into SW1990 and CAPAN-1 cells. Afterwards, cell lysates were harvested and incubated with Dynabeads M-280 Streptavidin (Sigma-Aldrich) in line with the manufacturer’s protocols. After washing with wash buffer (Invitrogen), RNA complexes were separated and purified with lysis buffer and proteinase K. Finally, purified RNA was analyzed by qRT-PCR.

### 2.13 Luciferase reporter assay

The fragments of wild-type (WT) and mutant (MUT) SLCO4A1-AS1 or KIF21B containing putative binding site of miR-4673 were synthesized and subcloned into pmirGLO vectors (Promega, Madison, WI, USA) to generate the recombinant reporters including SLCO4A1-AS1-WT, SLCO4A1-AS1-MUT, KIF21B-WT, and KIF21B-MUT. Next the reporters were co-transfected together with miR-4673 mimics, NC mimics, or miR-4673 mimics + pcDNA3.1/SLCO4A1-AS1 into PC cells. The luciferase activity after 48 h was evaluated by the Dual-Luciferase Reporter Assay System (Promega).

### 2.14 RIP assay

Magna RNA immunoprecipitation Kit (Millipore) was used for RIP assay. All the cell lysates were incubated with RIPA lysis buffer containing magnetic beads (Invitrogen) conjugated to antibodies of human anti-Ago2 (1:30, ab186733, Abcam) or control anti-IgG (1:16, ab182931, Abcam). The coprecipitated RNA was eluted from the beads and analyzed by PCR.

### 2.15 Statistical analysis

All experiments in the present study were repeated in triplicate. The data are expressed as the mean value ± SD and analyzed using SPSS 18.0 software (SPSS, Chicago, IL, USA). The differences of two or more groups were assessed by Student’s *t* test or one-way analysis of variance (ANOVA) followed by Tukey’s *post hoc* analysis, with *p* < 0.05 representing as statistically significant.

## 3 Results

### 3.1 Silencing SLCO4A1-AS1 inhibits the cellular processes of PC

To examine whether SLCO4A1-AS1 was dysregulated in PC, we first explored the expression profile of SLCO4A1-AS1 in PAAD from GEPIA database, and found that SLCO4A1-AS1 was upregulated in PAAD tissues compared to normal tissues (Figure 1a). Additionally, SLCO4A1-AS1 was overexpressed in PC cells in comparison to the normal H6C7 cells, as shown by qRT-PCR analysis (Figure 1b). Among the PC cell lines, SLCO4A1-AS1 expression in SW1990 and CAPAN-1 cells was the highest, thus they were singled out for the following experiments. To figure out the function of SLCO4A1-AS1 in PC, SW1990 and CAPAN-1 cells were transfected with sh-SLCO4A1-AS1#1/2 or sh-NC to measure the efficiency of SLCO4A1-AS1 knockdown. We discovered that SLCO4A1-AS1 expression displayed a significant decrease in selected cells in contrast to NC group (Figure 1c). Next we carried out CCK-8 assay and found that the silencing of SLCO4A1-AS1 repressed PC cell viability (Figure 1d). The findings of the colony formation assay also elucidated that SLCO4A1-AS1 downregulation attenuated cell proliferation (Figure 1e). Furthermore, the influence of SLCO4A1-AS1 depletion on cell apoptosis examined by flow cytometry and western blot analysis indicated that SLCO4A1-AS1 downregulation induced apoptosis in PC cells (Figure 1f and g). Subsequently, we conducted wound healing assay and discovered that SLCO4A1-AS1 depletion repressed cell migratory potential (Figure 1h). Later, the transwell assay demonstrated the repressed invasive ability of PC cells after the silencing of SLCO4A1-AS1 (Figure 1i). These findings elucidated that SLCO4A1-AS1 works as a cancer-promoting gene in PC cells.

**Figure 1:** Silencing SLCO4A1-AS1 inhibits the cellular processes of PC. (a) SLCO4A1-AS1 expression pattern in PAAD was revealed in the boxplot from GEPIA. (b) SLCO4A1-AS1 expression in PC cell lines in contrast with normal H6C7 cells was examined by qRT-PCR. (c) qRT-PCR investigated the interfering efficiency of SLCO4A1-AS1 in PC cells. (d) CCK-8 assay was used to detect PC cell viability affected by SLCO4A1-AS1 knockdown. (e) The effect of SLCO4A1-AS1 knockdown on CAPAN-1 and SW1990 cell proliferation was investigated by colony formation assay. (f and g) The apoptosis of PC cells transfected with sh-SLCO4A1-AS1 was analyzed by flow cytometry and western blot analysis. (h) Wound healing assay measured how downregulated SLCO4A1-AS1 affected cell migration. (i) Transwell assay detected the invasive capability of PC cells after SLCO4A1-AS1 depletion. All experiments were performed in triplicate. More images for replicates are provided in a supplementary file named Replicate images. *p < 0.05 and **p < 0.01.

### 3.2 SLCO4A1-AS1 acts as a molecular sponge of miR-4673

Increasing studies have illustrated that lncRNAs exert regulatory function in the malignant processes of tumors by acting as competing endogenous RNAs (ceRNAs) to sponge miRNAs [18]. Considering that the nuclear-cytoplasmic localization of lncRNAs plays an important part in the molecular mechanism, we first conducted the subcellular fractionation assay, which suggested that SLCO4A1-AS1 was mainly located in cytoplasm of PC cells (Figure 2a). Moreover, six putative downstream miRNAs interacting with SLCO4A1-AS1 were selected from database of DIANA (Figure 2b). Thereafter, the result of RNA pull-down suggested that miR-4673 and miR-876-3p were enriched in PC cells treated with SLCO4A1-AS1 probe-biotin (Figure 2c). Next the expression of miR-4673 and miR-876-3p in PC cells and normal cells was assessed by qRT-PCR, suggesting that miR-4673 was significantly downregulated in PC cells (Figure 2d). In addition, the results of qRT-PCR demonstrated that miR-4673 expression was elevated in PC cells transfected with miR-4673 mimics (Figure 2e). Later, we analyzed the binding site of miR-4673 on SLCO4A1-AS1 with the use of DIANA database (Figure 2f). Furthermore, the binding relation between SLCO4A1-AS1 and miR-4673 was further verified by luciferase reporter assay. The findings depicted that upregulated miR-4673 attenuated the luciferase activity of SLCO4A1-AS1-WT reporter vector, while the luciferase activity of SLCO4A1-AS1-MUT remained almost unchanged with miR-4673 overexpression (Figure 2g). Collectively, SLCO4A1-AS1 can directly sponge miR-4673.

**Figure 2:** miR-4673 is directly absorbed by SLCO4A1-AS1. (a) Subcellular fractionation assay determined the localization of SLCO4A1-AS1 in PC cells. (b) We searched the downstream miRNAs of SLCO4A1-AS1 from the DIANA database. (c) RNA pull-down investigated the expression of candidate miRNAs pulled down by SLCO4A1-AS1 probe-biotin in PC cells. (d) The levels of selected miRNAs in PC cells were measured through qRT-PCR. (e) The overexpression efficiency of miR-4673 was subjected to qRT-PCR. (f) The binding site of SLCO4A1-AS1 on miR-4673 is revealed from DIANA database. (g) Luciferase reporter assay was employed to examine the luciferase activity of SLCO4A1-AS1-WT and SLCO4A1-AS1-MUT in PC cells transfected with miR-4673 mimics. All experiments were performed in triplicate. **p < 0.01.

### 3.3 Inhibition of miR-4673 reverses the effects of SLCO4A1-AS1 silencing on the phenotypes of PC cells

Subsequently, we investigated whether miR-4673 inhibition had an effect on the carcinogenic role of SLCO4A1-AS1 in PC. As shown by qRT-PCR, miR-4673 was significantly downregulated in miR-4673 inhibitors-transfected CAPAN-1 and SW1990 cells (Figure 3a). The results from CCK-8 assay demonstrated that miR-4673 inhibitors significantly attenuated SLCO4A1-AS1 knockdown-induced suppression of PC cell viability (Figure 3b). Similarly, colony formation assay showed that SLCO4A1-AS1 knockdown led to a significant reduction in the number of colonies of CAPAN-1 and SW1990 cells; however, treatment of miR-4673 inhibitors was shown to alleviate this effect (Figure 3c), indicating that miR-4673 inhibitors might have a promotive effect on cell proliferation. As displayed by Figure 3d and e, SLCO4A1-AS1 silencing-induced cell apoptosis was partially reversed by miR-4673 inhibitors in CAPAN-1 and SW1990 cells. Furthermore, miR-4673 inhibition rescued the decrease in the migratory and invasive abilities of PC cells which was caused by SLCO4A1-AS1 silencing, as shown by wound healing and transwell assays (Figure 3f and g). Hence, inhibition of miR-4673 can reverse SLCO4A1-AS1 knockdown-mediated suppressive effects on the malignant phenotypes of PC cells.

**Figure 3:** miR-4673 inhibition reverses SLCO4A1-AS1 knockdown-induced suppressive effects on the phenotypes of PC cells. (a) qRT-PCR analysis for detecting the transfection efficiency of miR-4673 inhibitors in CAPAN-1 and SW1990 cells. (b) The viabilities of CAPAN-1 and SW1990 cells transfected with sh-NC, sh-SLCO4A1-AS1#1, or sh-SLCO4A1-AS1#1 + miR-4673 inhibitors were analyzed by CCK-8 assay. (c) Colony formation assay was used to examine the proliferation of PC cells with above transfection. (d and e) The apoptosis of transfected PC cells was assessed by flow cytometry and western blot analysis. (f and g) Wound healing and transwell assays were performed to evaluate the migration and invasion of PC cells with above transfection. All experiments were performed in triplicate. More images for replicates are provided in a supplementary file named Replicate images. **p < 0.01.

### 3.4 KIF21B is a target gene for miR-4673

We next screened out eight candidate messenger RNAs (mRNAs) targeted by miR-4673 with TargetScan database (Figure 4a). PCR analysis demonstrated that three mRNAs (KIF21B, KREMEN1, and FBXL18) were markedly downregulated in PC cells after upregulating miR-4673 (Figure 4b). Next the level of KIF21B was enhanced in PC cells among three mRNAs, as illustrated by qRT-PCR (Figure 4c). The protein level of KIF21B was decreased in PC cells upon miR-4673 overexpression, as indicated by western blot analysis (Figure 4d). Additionally, silencing SLCO4A1-AS1 led to a significant reduction in both mRNA and protein levels of KIF21B in PC cells (Figure 4e). Afterwards, the binding site of miR-4673 on KIF21B 3′-UTR was predicted by TargetScan database (Figure 4f). Moreover, qRT-PCR showed that SLCO4A1-AS1 was upregulated in CAPAN-1 and SW1990 cells after transfection of pcDNA3.1/SLCO4A1-AS1 (Figure 4g). Later, the relationship among SLCO4A1-AS1, miR-4673, and KIF21B was detected by luciferase reporter assay, which demonstrated that the luciferase activity of KIF21B-WT was attenuated by miR-4673 upregulation and then enhanced by SLCO4A1-AS1 overexpression in SW1990 and CAPAN-1 cell lines, while the luciferase activity of KIF21B-MUT witnessed no significant change (Figure 4h). Besides, the RIP assay examined the interaction of SLCO4A1-AS1, miR-4673, and KIF21B, indicating their co-existence in the RNA-induced silencing complex (RISC) (Figure 4i). Additionally, the data from GEPIA database reveal the upregulation of KIF21B in PAAD tissues (Figure 4j). These findings elucidated that KIF21B is the downstream target for miR-4673, and SLCO4A1-AS1 upregulates KIF21B expression at a miR-4673 dependent way.

**Figure 4:** KIF21B is targeted by miR-4673. (a) The eight candidate mRNAs of miR-4673 were selected from TargetScan database. (b) qRT-PCR analyzed the expression of these miRNAs in PC cells transfected with miR-4673 mimics. (c) The expression of selected mRNAs in PC cells were detected through qRT-PCR. (d) The protein level of KIF21B in PC cells after miR-4673 upregulation was analyzed by qRT-PCR. (e) qRT-PCR assessed both the mRNA and protein levels of KIF21B in PC cells after silencing SLCO4A1-AS1. (f) We searched the binding site of KIF21B on miR-4673 from TargetScan database. (g) The overexpression efficiency of SLCO4A1-AS1 in PC cells was measured through qRT-PCR. (h) Luciferase reporter assay detected the luciferase activity of KIF21B-WT and KIF21B-MUT in PC cells transfected with miR-4673 mimics or miR-4673 mimics + pcDNA3.1/SLCO4A1-AS1. (i) RIP assay was applied to confirm the co-existence of SLCO4A1-AS1, miR-4673, and KIF21B in RISC. (j) The expression of KIF21B in PAAD and normal tissues is shown by GEPIA database. All experiments were performed in triplicate. *p < 0.05 and **p < 0.01.

### 3.5 SLCO4A1-AS1 positively modulates the malignant progression of PC cells via upregulating KIF21B

To further expose the functional mechanism of SLCO4A1-AS1 in PC cells, rescue assays were carried out. First, qRT-PCR depicted that KIF21B expression was increased in PC cells transfected with pcDNA3.1/KIF21B (Figure 5a). Next as indicated by CCK-8 assay, SW1990 and CAPAN-1 cell viabilities reduced by the depletion of SLCO4A1-AS1 were reversed by overexpressed KIF21B (Figure 5b). In addition, the results of colony formation assay depicted that the SLCO4A1-AS1 silence-mediated decrease in proliferative ability of PC cells was countervailed by the upregulation of KIF21B (Figure 5c). Flow cytometry and western blot analysis elucidated that enhanced KIF21B expression offset the apoptosis rate of PC cells formerly increased by SLCO4A1-AS1 downregulation (Figure 5d and e). Furthermore, the suppressive influence of SLCO4A1-AS1 downregulation on PC cell migratory capacity was rescued by the overexpression of KIF21B as shown by wound healing assay (Figure 5f). Later, the result of transwell assay indicated the counteracting impact of upregulated KIF21B on the inhibited cell invasion of SW1990 and CAPAN-1 cells caused by the knockdown of SLCO4A1-AS1 (Figure 5g). These data illustrated that SLCO4A1-AS1 upregulates KIF21B expression by competitively interacting with miR-4673, thereby modulating the malignant behaviors of PC cells.

**Figure 5:** SLCO4A1-AS1 accelerates the cellular process of PC through regulating KIF21B. (a) qRT-PCR detected the overexpression efficiency of KIF21B in PC cells. (b) CCK-8 assay was carried out to investigate the impact of upregulated KIF21B on suppressed cell viability caused by depleting SLCO4A1-AS1. (c) The SLCO4A1-AS1 silence-reduced proliferation capacity of PC cells was affected by KIF21B overexpression, as indicated by colony formation assay. (d and e) The apoptosis of PC cells transfected with appointed plasmids was analyzed by flow cytometry and western blot analysis. (f) The influence of SLCO4A1-AS1 knockdown on KIF21B overexpression-enhanced migrated capability of PC cells was determined by wound healing assay. (g) The change in invasive capability of PC cells with designated transfections was investigated by Transwell assay. All experiments were performed in triplicate. More images for replicates are provided in a supplementary file named Replicate images. **p < 0.01.

## 4 Discussion

As one prevalent in digestive malignancy with high morbidity and mortality, PC has imposed tremendous pressure on public health [19]. Moreover, despite new technologies and therapies for early diagnosis, most patients are still diagnosed at an advanced stage for the insidious onset of this disease [20]. Unfortunately, these patients are unlikely subject to radical resection, and adjuvant chemotherapy has limited influence because of the type and efficacy [21]. Hence, there is an exigent need to figure out novel and effective biomarkers to improve the prognosis of PC. Previous studies have revealed that the aberrant expression of lncRNAs plays a pivotal role in regulating the malignant properties of PC. For instance, lncRNA nuclear paraspeckle assembly transcript 1 facilitates the tumorigenesis and growth of PC via stabilizing E74 like ETS transcription factor 3 [22]. LncRNA 00976 upregulates OTU deubiquitinase 7B to enhance PC cell growth and invasion by binding with miR-137 [23]. LINC01559 facilitates PC cell proliferation and migration through Yes1 associated transcriptional regulator-mediated pathway [24]. Nevertheless, the role of SLCO4A1-AS1 in the biological mechanism of PC remains unclear. Herein we confirmed that SLCO4A1-AS1 was overexpressed in PC. Additionally, SLCO4A1-AS1 downregulation repressed cell growth and motion, and stimulated cell apoptosis of PC, indicating that SLCO4A1-AS1 exerted oncogenic functions in PC.

It has been elucidated that lncRNAs serve as ceRNAs by performing as molecular sponges of miRNAs, thereby regulating the specific target genes for miRNAs [25]. For instance, lncRNA LINC01559 promotes the cellular process of PC by sponging miR-1343-3p to upregulate Raf-1 proto-oncogene, serine/threonine kinase level [26]. In our study, the specific miR-4673 sponged by SLCO4A1-AS1 was selected with bioinformatic tools. miR-4673 was reported as a tumor suppressor in hepatocellular carcinoma [27]. Presently, we verified that the miR-4673 was downregulated in PC cells. Moreover, the binding relation between SLCO4A1-AS1 and miR-4673 was detected. Inhibition of miR-4673 was shown to reverse SLCO4A1-AS1 knockdown-mediated inhibitory effects on the malignant behaviors of PC cells. Therefore, miR-4673 can directly interact with SLCO4A1-AS1.

Subsequently, KIF21B, as the downstream gene for miR-4673, was screened out from TargetScan database. KIF21B belongs to the motor of Kinesin-4 motor and is located at 1q32.1 [28]. Previous studies validated that KIF21B, a classic kinesin protein, was able to regulate microtubule dynamics [29]. It is widely known that kinesin proteins and microtubules exert pivotal functions in tumor progression intercellular and signal transduction [30]. It was reported that KIF21B exhibited a carcinogenic function in non-small cell lung cancer; silencing KIF21B represses cell growth and induces apoptosis [28]. Furthermore, KIF21B is overexpressed and facilitates cellular behaviors in hepatocellular carcinoma [31]. In the current study, we verified the overexpression of KIF21B and the binding capacity between miR-4673 and KIF21B in PC cells. Furthermore, the repressed cellular processes of PC by depleting SLCO4A1-AS1 was rescued with the upregulation of KIF21B.

In summary, we identified SLCO4A1-AS1 as a cancer-causing gene, exerting critical functions in cellular processes of PC. Mechanistically, SLCO4A1-AS1, as a ceRNA, upregulates KIF21B to positively modulate the molecular processes of PC via sponging miR-4673. These results showed that SLCO4A1-AS1/miR-4673/KIF21B axis might be an effective biomarker for the prognosis of PC, deepening the understanding of its pathogenesis. Other possible molecules involved in SLCO4A1-AS1-mediated ceRNA network require further investigation. For example, miR-223-3p and miR-335-5p were reported to a downstream molecule of SLCO4A1-AS1 involved in non-small-cell lung cancer and bladder cancer, respectively [13,15]. Additionally, miR-223-3p was reported to be upregulated in the serum of PC and miR-335-5p was shown to be sponged by LINC00941 and involved in the progression of PC [32,33]. More studies are needed to be carried out in the future.

## Abbreviations

CCK-8: cell counting kit-8
cDNA: complementary DNA
ceRNA: competing endogenous RNA
DMEM: Dulbecco’s modified eagle’s medium
KIF21B: kinesin family member 21B
lncRNAs: long non-coding RNAs
NC: negative control
mRNA: messenger RNA
miR-4673: microRNA-4673
MUT: mutant
PAAD: pancreatic adenocarcinoma
PC: pancreatic cancer
PI: propidium iodide
PVDF : polyvinylidene fluoride
qRT-PCR : quantitative real-time PCR
RIPA : RNA immunoprecipitation assay
SDS-PAGE : sodium dodecyl sulfate polyacrylamide gel electrophoresis
shRNAs : short-hairpin RNAs
SLCO4A1-AS1: lncRNA solute carrier organic anion transporter family member 4A1 antisense RNA 1
V-FITC : V-fluorescein isothiocyanate
WT: wild type
